The article "Construction and Bioinformatics Analysis of the miRNA-mRNA Regulatory Network in Diabetic Nephropathy" was retracted in 2023. Reasons: signs of a paper mill; suspected computer-generated content; unreliable results or conclusions; concerns about the data.

# Construction and Bioinformatics Analysis of the miRNA-mRNA Regulatory Network in Diabetic Nephropathy

**DOI:** 10.1155/2021/8161701

**Published:** 2021-11-18

**Authors:** Yameng Li, Yukun Xu, Yawei Hou, Rui Li

**Affiliations:** ^1^School of Traditional Chinese Medicine, Shandong University of Traditional Chinese Medicine, Shandong 250014, China; ^2^Department of Geriatrics, Affiliated Hospital of Shandong University of Traditional Chinese Medicine, Shandong, China

## Abstract

**Background:**

MicroRNA (miRNA) has been confirmed to be involved in the occurrence, development, and prevention of diabetic nephropathy (DN), but its mechanism of action is still unclear.

**Objective:**

With the help of the GEO database, bioinformatics methods are used to explore the miRNA-mRNA regulatory relationship pairs related to diabetic nephropathy and explain their potential mechanisms of action.

**Methods:**

The DN-related miRNA microarray dataset (GSE51674) and mRNA expression dataset (GSE30122) are downloaded through the GEO database, online analysis tool GEO2R is used for data differential expression analysis, TargetScan, miRTarBase, and miRDB databases are used to predict potential downstream target genes regulated by differentially expressed miRNAs, and intersection with differential genes is used to obtain candidate target genes. According to the regulatory relationship between miRNA and mRNA, the miRNA-mRNA relationship pair is clarified, and the miRNA-mRNA regulatory network is constructed using Cytoscape. DAVID is used to perform GO function enrichment analysis and KEGG pathway analysis of candidate target genes. By GeneMANIA prediction of miRNA target genes and coexpressed genes, the protein interaction network is constructed. *Results and Conclusion*s. A total of 67 differentially expressed miRNAs were screened in the experiment, of which 42 were upregulated and 25 were downregulated; a total of 448 differentially expressed mRNAs were screened, of which 93 were upregulated and 355 were downregulated. Using TargetScan, miRTarBase, and miRDB databases to predict downstream targets of differentially expressed miRNAs, 2283 downstream target genes coexisting in 3 databases were predicted to intersect with differentially expressed mRNAs to obtain 96 candidate target genes. Finally, 44 miRNA-mRNA relationship pairs consisting of 12 differentially expressed miRNAs and 27 differentially expressed mRNAs were screened out; further analysis showed that miRNA regulatory network genes may participate in the occurrence and development of diabetic nephropathy through PI3K/Akt, ECM-receptor interaction pathway, and RAS signaling pathway.

## 1. Introduction

In recent years, impaired glucose tolerance and diabetes incidence was on the rise every year, in 2017, about 425 million people worldwide suffer from diabetes, and the prevalence rate is about 8.4%. In 2045, the global diabetes is expected to increase to 629 million people, about 9.9% [1]. In China, the 2013 prevalence rate was 10.9%, and prediabetes was 35.7% [2]. In developed countries, diabetic nephropathy (DN) is the main cause of end-stage renal disease. In developing countries, with the improvement of the economic level and the change of people's living habits, DN is rapidly replacing primary glomerular disease and becoming the main cause of end-stage kidney disease. A recent cross-sectional study in my country showed that about 4.5% of hospitalized patients (1.8 million) were identified as CKD, and the proportion increased from 3.7% in 2010 to 4.7% in 2015. From 2010 to 2015, the incidence of DN and hypertensive nephropathy showed an upward trend (19.5% and 24.3% and 11.5% and 15.9%, respectively), especially among residents in northern Chinese cities [3]. In addition, DN has also become one of the main causes of end-stage renal disease in my country (accounting for 16.4%), and it is increasing year by year [4].

The pathogenesis of DN is complex, but current studies have confirmed that miRNA plays an extremely important role in the development of DN. There are few studies on miRNA-mRNA regulatory networks. This experiment intends to use the DN-related mRNA and miRNA datasets in the GEO database to construct an miRNA-mRNA regulatory network, explore its mechanism of action, and provide an important theoretical reference and scientific basis for early diagnosis and targeted therapy of DN.

## 2. Materials and Methods

### 2.1. Design: Molecular Bioinformatics Research

#### 2.1.1. Source of Information

The microarray data of the miRNA expression profile and mRNA expression profile related to DN are retrieved from the GEO (Gene Expression Omnibus) database of NCBI. The screening criteria are kidney samples from DN patients and healthy people, and cell lines or animal models are excluded. Finally, download the miRNA expression data set GSE51674 and mRNA expression data set GSE30122 that meet the requirements. The dataset GSE51674 is based on the platform GPL10656 and contains 16 kidney tissue samples, including 6 DN patients, 4 males and 2 females, with an average age of 59 years. The average age of 4 patients in the healthy group was 38 years, 3 males and 1 female; the dataset GSE30122 was based on the platform GPL571 and contained 69 kidney tissue samples. 26 healthy glomerular samples were selected as the control group and 9 DN glomerular sample cases as the disease group.

### 2.2. Methods

#### 2.2.1. Data Processing and Differential Expression Analysis

GEO online analysis tool GEO2R (https://www.ncbi.nlm.nih.gov/geo/geo2r/) is used to obtain differential mRNA and miRNA and then screened for differential genes. The screening standard is set as adj. *p*. val<0.01 and |log2 fold change (FC)| >1. A volcano map and a cluster map were constructed to visualize the differential expression data.

#### 2.2.2. Target Gene Prediction and miRNA-mRNA Regulatory Network Construction

According to differential miRNA obtained from the analysis of the dataset GSE51674, the downstream target gene prediction is performed through the TargetScan [5], miRTarBase [6], miRDB [7, 8] databases, and the downstream target genes predicted by the three databases, at the same time, are compared with the dataset. GSE30122 differentially expressed mRNA takes the intersection to obtain candidate target genes. With the help of the regulatory relationship between miRNA and mRNA, an miRNA-mRNA regulatory network is established. Cytoscape [9] software (version 3.7.2) is used to visualize the miRNA-mRNA regulatory network.

#### 2.2.3. External Validation Was Performed with the Validation Datasets

The DN-related mRNA expression dataset GSE30528 was downloaded from the GEO database. GSE30528 is based on the platform GPL571, which contains 22 glomerular samples, 9 cases of DN glomeruli and 13 cases of normal glomeruli. By intersecting the differentially expressed mRNAs analyzed by GSE30528 and GSE30122, cross-validation of common genes in the development of DN was performed.

#### 2.2.4. Candidate Target Gene GO Function and KEGG Pathway Enrichment Analysis

For better understanding these screened candidate target genes, DAVID [10] was utilized to perform GO function and KEGG pathway enrichment analysis.

#### 2.2.5. Construction of the miRNA-Regulated Target Gene-Protein Interaction Network and Prediction of Coexpressed Genes

The PPI network was constructed, and its coexpression relationship with miRNA genes was determined using the GeneMANIA [11] plugin of Cytoscape software.

## 3. Results

### 3.1. Differentially Expressed miRNAs

In the GSE51674 dataset, the kidney tissues of healthy individuals are compared with the kidney tissue samples of DN patients to obtain 67 miRNAs that are differentially expressed, up 42 （hsa-miR-135b, hsa-miR-126^*∗*^, hsa-miR-150, hsa-miR-146b-5p, hsa-miR-142-3p, hsa-miR-186, hsa-miR-142-5p, hsa-miR-374a, hsa-miR-146a, hsa-miR-374b, hsa-miR-223, hsa-miR-95, hsa-miR-34a, hsa-miR-199a-5p, hsa-miR-155, hsa-miR-376c, hsa-miR-335, hsa-miR-199b-5p, hsa-miR-301a, hsa-miR-132, hsa-miR-31^*∗*^, hsa-miR-139-5p, hsa-miR-31, hsa-miR-377, hsa-miR-181c, hsa-miR-429, hsa-miR-361-3p, hsa-miR-454, hsa-miR-505, hsa-miR-590-5p, hsa-miR-183, hsa-miR-145^*∗*^, hsa-miR-21, hsa-miR-28-5p, hsa-let-7a, hsa-miR-195, hsa-miR-16, hsa-let-7f, hsa-let-7g, hsa-miR-130a, hsa-miR-126, and hsa-let-7b） and down 25 （hsa-miR-138, hsa-miR-625^*∗*^, hsa-miR-1227, hsa-miR-1307, hsa-miR-339-3p, hsa-miR-563, hsa-miR-92b, hsa-miR-1274b, hsa-miR-320a, hsa-miR-634, hsa-miR-1229, hsa-miR-1539, hsa-miR-2116^*∗*^, hsa-miR-296-5p, hsa-miR-602, hsa-miR-1275, hsa-miR-572, hsa-miR-1280, hsa-miR-940, hsa-miR-1268, hsa-miR-1234, hsa-miR-1228, hsa-miR-1225-3p, hsa-miR-33b^*∗*^, and hsa-miR-1237）. A heatmap and volcano map were plotted through http://www.bioinformatics.com.cn, a free online platform for data analysis and visualization (Figures 1 and 2).

### 3.2. Differentially Expressed mRNAs

Compared with healthy glomerular samples in the dataset GSE30122, DN glomerular samples obtained 448 differentially expressed genes, of which 93 were upregulated and 355 were downregulated. The top 58 differential genes with the larger absolute value of the difference multiple to the cluster are selected (Figures 3 and 4).

### 3.3. Target Gene Prediction and Regulatory Network Construction

TargetScan, miRTarBase, and miRDB databases were used to predict the downstream targets of differentially expressed miRNAs. Among them, 2283 mRNAs existed in three databases at the same time (Figure 5(a)), and 1077 miRNA-mRNA relationship pairs existed in 3 databases at the same time. The three databases exist in the differentially expressed genes and genes on the intersection to obtain 96 candidate target genes (Figure 5(b)).

According to the negative regulatory relationship between miRNA and mRNA, 44 miRNA-mRNA relationship pairs consisting of 12 differentially expressed miRNAs and 27 differentially expressed mRNAs were finally screened out. Cytoscape software was used to visualize the miRNA-mRNA regulatory network (Figure 6 and Table 1).

### 3.4. External Validation Was Performed with the Validation Datasets

The dataset GSE30528 was screened for differential genes, and the screening criteria were set as adj. *p*. val<0.01 and |log2 fold change (FC)| >1. 372 differential genes were screened out, of which 304 were downregulated and 68 were upregulated. Compared with the GSE30122 data, it can be seen that all 50 differential genes are upregulated (Figure 7(a)), and 273 differential genes are all downregulated (Figure 7(b)).

### 3.5. Functional Enrichment of Candidate Target Genes and KEGG Analysis

GO function and KEGG pathway enrichment analyses of candidate target genes were performed based on DAVID. The BP analysis showed vasculogenesis, heart development, extracellular matrix organization, ventricular septum morphogenesis, positive regulation of cell migration, positive regulation of transcription, DNA template, cell-matrix adhesion, transforming growth factor-beta receptor signaling pathway, negative regulation of cell migration, cell migration, sex determination, and commissural neuron axon guidance (Figure 8). The 13 enrichment pathways that resulted from KEGG pathway analysis were focal adhesion, arrhythmogenic right ventricular cardiomyopathy (ARVC), platelet activation, hypertrophic cardiomyopathy (HCM), proteoglycans in cancer, dilated cardiomyopathy, PI3K-Akt signaling pathway, adherens junction, Rap1 signaling pathway, regulation of the actin cytoskeleton, pathways in cancer, RAS signaling pathway, and ECM-receptor interaction (Figure 9).

### 3.6. Construction of the miRNA-Regulated Target Gene-Protein Interaction Network and Prediction of Genes Coexpressed with Differential mRNA

The GeneMANIA plugin in Cytoscape software was used to construct miRNA-regulated target gene-protein interaction relationships and predict genes coexpressed with differential mRNAs (Figure 10).

## 4. Discussion

DN is the main microvascular complication of diabetes. In 2015, diabetes-related chronic kidney disease patients in China accounted for 1.10% of the total hospitalized population, surpassing primary glomerulonephritis-related chronic kidney disease patients (0.75%), becoming one of the main causes of chronic kidney disease [12]. In Western countries, DN is leading to end-stage renal disease (ESRD) which is the primary factor. With the rapid increase in the incidence of diabetes, the personal and socioeconomic burden caused by DN is very heavy. Moreover, the time for DN patients to start renal replacement therapy is earlier than that of other kidney disease patients, and it greatly affects the patient's quality of life. Moreover, once the patient develops a large amount of proteinuria, there is no effective treatment plan. This suggests that the discovery of the molecular mechanism of DN is essential for the treatment and prevention of DN.

Studies have found that many miRNAs have been proven to promote DN development or reduce DN damage. miR-27a [13] activates TGF-*β*/Smad3 signaling by inhibiting PPAR*γ* and promotes connective tissue growth factor (CTGF), fibronectin, and collagen. Changes in the expression of protein I promote the deterioration of tubular interstitial fibrosis in DN and accelerate the progression of DN. miR-218 [14] accelerates podocyte apoptosis induced by high glucose by directly downregulating HO-1 and promoting p38-MAPK activation. miR346 [15] participates in the epithelial-mesenchymal transition of mouse podocytes under high glucose conditions, and miR-346 can indirectly regulate the expression of GSK-3*β* in mouse podocytes and play a renal protective role. miR-34c [16] overexpression inhibits the Notch signaling pathway by targeting Notch1 and Jaggged1 in podocytes treated with high glucose, thereby inhibiting podocyte apoptosis induced by high glucose and reducing DN kidney damage. miR-146a [17] can prevent diabetic glomerulopathy and podocyte damage by inhibiting ErbB4/EGFR.

In this experiment, we used GEO dataset GSE30122 to obtain 448 differentially expressed genes, of which 93 were upregulated and 355 were downregulated. The miRNA expression dataset GSE51674 analyzed, screened, and obtained 67 miRNAs that were differentially expressed, 42 upregulated miRNAs and 25 downregulated miRNAs. Using TargetScan, miRTarBase, and miRDB databases to predict downstream targets of differentially expressed miRNAs, 2283 mRNAs existed in three databases at the same time, and 1077 miRNA-mRNA relationship pairs existed in 3 databases at the same time. Intersection of genes and differential genes that exist in three databases at the same time obtained 96 candidate target genes. According to the negative regulatory relationship between miRNA and mRNA, 44 miRNAs consisting of 12 differentially expressed miRNAs and 27 differentially expressed mRNAs are finally screened out. These different miRNAs and mRNAs may be the key nodes in the occurrence and development of DN.

The KEGG pathway enrichment analysis of candidate target genes revealed that it is related to 13 signaling pathways, among which the phosphatidyl inositol 3-kinase (PI3K)/protein kinase B (AKT) signaling pathway is one of the classic cancer signal transduction pathways. The phosphatidyl inositol 3-kinase (PI3K)/protein kinase B (AKT) signaling pathway is a hot spot for cancer molecular biomarkers and targeted therapy. Studies have found that [18] notoginsenoside R1 (NR1) inhibits inflammation and apoptosis through the PI3K/Akt signaling pathway to improve podocyte damage in a rat model of diabetic nephropathy. Zang et al. [19] found that by inhibiting the PI3K-Akt pathway, it can inhibit the proliferation of mesangial cells and the accumulation of the extracellular matrix in the rat diabetic model, thereby exerting renal protection. Glomerular mesangial cells are essential for maintaining and regulating glomerular filtration. The abnormal proliferation of glomerular mesangial cells leads to the accumulation of the mesangial extracellular matrix (ECM), which further promotes glomerular dysfunction and kidney disease. Studies have found that inhibiting the ECM-receptor interaction pathway can reduce the ability of human renal mesangial cell damage caused by advanced glycation end products, thereby inhibiting the development of DN [20]. The activation of the renin-angiotensin system (RAS) is one of the main risk factors for progressive chronic kidney disease. Studies have found that RAS activation can accelerate the progression of glomerulosclerosis [21].

Although this experiment has constructed a potential miRNA-mRNA regulatory network based on bioinformatics, it still has certain limitations. The glomerular samples of DN in the experiment come from patients with DN at different stages, and there is no distinction between the renal glomeruli of DN at different stages. DN has a small sample of glomeruli. The sample source of differential miRNA is whole kidney tissue, and the sample source of differential mRNA is the glomerulus. And there is no design of blood, urine, and other samples. The source of blood and urine samples will more accurately explain the physiological and pathological process of DN. And this experiment only involves chip sequencing data, not included in the high-throughput sequencing dataset. In summary, DN is the result of the joint action of multiple pathogenesis. The experiment integrated and analyzed differentially expressed miRNA and mRNA in DN kidney tissue and successfully constructed an miRNA-mRNA regulatory network. 44 miRNA-mRNA relationship pairs were composed of 12 differentially expressed miRNAs and 27 differentially expressed mRNAs. These differential miRNAs and mRNAs may be the key nodes in the occurrence and development of the DN disease. It provides new ideas for the pathogenesis and treatment of DN. However, this study still needs to be verified by further animal experiments.

## Figures and Tables

**Figure 1:** Differentially expressed miRNA levels in kidney tissue samples from healthy individuals and diabetic nephropathy patients. Red represents upregulation, and green represents downregulation.

**Figure 2:** Volcano map of miRNAs differently expressed in DN. Red dots represent upregulation, blue dots represent downregulation, and gray dots represent no differential expression.

**Figure 3:** The top 58 differential genes with the larger absolute value of the fold change. Red represents upregulation, and green represents downregulation.

**Figure 4:** Volcano map of mRNAs differently expressed in DN. Red dots represent upregulation, blue dots represent downregulation, and gray dots represent no differential expression.

**Figure 5:** Screening of target genes. (a) Venn diagram of TargetScan, miRTarBase, and miRDB databases predicting miRNAs corresponding to downstream target genes. (b) Venn diagram of differentially expressed mRNA and miRNA downstream target genes.

**Figure 6:** DN-related miRNA-mRNA regulatory network. Red indicates downregulation, and blue indicates upregulation. V-type and circle indicate miRNA and mRNA, respectively.

**Figure 7:** External dataset cross-validation Venn diagram.

**Figure 8:** Biological process enrichment analysis of candidate target genes.

**Figure 9:** KEGG pathway analysis was performed for the candidate target genes.

**Figure 10:** The coexpression network is displayed after the differential mRNA analysis of miRNA regulation by GeneMANIA plugin. *Note.* The black circle represents differential mRNA regulated by miRNA, gray circles represent coexpressed differential mRNAs, and the circle size represents the degree of genes in the correlation network.

**Table 1:** |miRNA-mRNA regulatory relationships.

miRNA	miRNA logFC	mRNA	mRNA logFC
hsa-let-7f	1.43	TGFBR3	−1.7269436
hsa-let-7f	1.43	GALC	−1.51748262
hsa-let-7f	1.43	ELF4	−1.03535741
hsa-miR-130a	1.3	GJA1	−1.67408832
hsa-miR-130a	1.3	DLC1	−1.52540045
hsa-miR-130a	1.3	JARID2	−1.36120294
hsa-miR-130a	1.3	TGFBR2	−1.33524188
hsa-miR-130a	1.3	CAMSAP2	−1.20387513
hsa-miR-130a	1.3	QKI	−1.10281385
hsa-miR-130a	1.3	DLG5	−1.00837835
hsa-miR-132	3.8	CAMSAP2	−1.20387513
hsa-miR-142-5p	5.37	ROBO1	−1.6019278
hsa-miR-142-5P	5.37	ACTN4	−1.09424855
hsa-miR-145^*∗*^	2.82	ITGB8	−1.79039728
hsa-miR-145^*∗*^	2.82	SERINC5	−1.47588306
hsa-miR-145^*∗*^	2.82	ANKRD28	−1.1428612
hsa-miR-145^*∗*^	2.82	ERG	−1.72463362
hsa-miR-145^*∗*^	2.82	NEDD9	−1.08024948
hsa-miR-145^*∗*^	2.82	TGFBR2	−1.33524188
hsa-miR-145^*∗*^	2.82	PHACTR2	−1.07106447
hsa-miR-145^*∗*^	2.82	CTNNBIP1	−1.62905063
hsa-miR-145^*∗*^	2.82	PODXL	−1.33174404
hsa-miR-223	4.57	F3	−1.56187542
hsa-miR-301a	3.81	DLC1	−1.52540045
hsa-miR-301a	3.81	JARID2	−1.36120294
hsa-miR-301a	3.81	TGFBR2	−1.33524188
hsa-miR-301a	3.81	CAMSAP2	−1.20387513
hsa-miR-301a	3.81	QKI	−1.10281385
hsa-miR-301a	3.81	DLG5	−1.00837835
hsa-miR-31^*∗*^	3.75	TBXA2R	−1.91556976
hsa-miR-429	3.35	ZEB1	−1.54067522
hsa-miR-429	3.35	QKI	−1.10281385
hsa-miR-429	3.35	DLC1	−1.52540045
hsa-miR-429	3.35	VEGFA	−2.15367902
hsa-miR-429	3.35	CAMSAP2	−1.20387513
hsa-miR-429	3.35	ZFPM2	−1.3592116
hsa-miR-454	3.09	DLC1	−1.52540045
hsa-miR-454	3.09	JARID2	−1.36120294
hsa-miR-454	3.09	TGFBR2	−1.33524188
hsa-miR-454	3.09	CAMSAP2	−1.20387513
hsa-miR-454	3.09	QKI	−1.10281385
hsa-miR-454	3.09	DLG5	−1.00837835
hsa-miR-590-5p	2.84	RECK	−1.56182514
hsa-miR-92b	-2.22	SOX4	1.04266344

## Data Availability

The simulation experiment data used to support the findings of this study are available from the corresponding author upon request.
